# Rare Case of Tubercular Serpiginous-Like Choroiditis

**DOI:** 10.7759/cureus.57093

**Published:** 2024-03-27

**Authors:** Renu Magdum, Tushar Agrawal, Deepaswi Bhavsar, Nilesh Giri, Ozukhil Radhakrishnan

**Affiliations:** 1 Ophthalmology, Dr. D. Y. Patil Medical College, Hospital and Research Centre, Pune, IND

**Keywords:** tuberculosis (tb), white dot syndrome, bilateral uveitis, macula, serpiginous-like choroiditis

## Abstract

Serpiginous choroiditis is a rare cause of posterior uveitis, included in the spectrum of white dot syndromes. It occurs as a result of an autoimmune process but could be associated with infections such as tuberculosis (TB) (serpiginous-like choroiditis). Tubercular serpiginous-like choroiditis is more commonly reported in Southeast Asian countries than in Western countries. We report a case of an Indian male in his late 30s with bilateral grey-yellowish subretinal infiltrates at the level of choroid with active scalloped edges having a positive TB-QuantiFERON Gold test (Cellestis Limited, Carnegie, Australia), who responded well to the treatment of intravenous methylprednisolone and systemic steroids (given initially to control the acute inflammation) while on anti-tubercular (anti-TB) therapy. The lesions finally completely healed on the anti-TB therapy.

## Introduction

Tuberculosis (TB) is an airborne communicable disease that most commonly involves the lungs. Up to 60% of people with extrapulmonary TB evidence may not have had pulmonary TB diagnosed; ocular TB may not always be linked to clinical evidence of pulmonary TB. Generally, the most prevalent symptoms related to eyes-and sometimes the only ones mentioned-are light sensitivity and hazy vision. Patients may present with anterior or posterior uveitis, choroid tubercles, retinal TB, orbit involvement, eyelid abscess, dacryoadenitis, subconjunctival nodules, or other complaints such as headache, flashes, floaters, or redness of the eye. Scleral inflammation with keratoconjunctivitis [1].

Serpiginous choroiditis belongs to a spectrum of diseases known as white dot syndromes. It has been reported that serpiginous-like choroiditis can have tuberculous involvement. The clinicopathologic correlation in tubercular serpiginous-like choroiditis remains unknown, despite the fact that histologic features in typical serpiginous choroiditis have been published. The diagnosis remains clinical. According to this study and past findings, it usually affects young to middle-aged persons from TB-endemic areas.

In this current investigation, the majority of eyes with serpiginous choroiditis had an initial lesion surrounding the optic nerve hypoplasia (ONH), a finding [2] that is common to other Indian and Caucasian studies. However, Abrez et al. showed [3] isolated macular involvement at a lower frequency (11% vs. 21%). A final visual acuity of less than 20/200 in up to 25% of eyes despite therapy was experienced by up to 75% of the patients because of numerous recurrences and the creation of new areas of choriocapillaris atrophy. In 1988, Mansour et al. reported [4] on seven eyes in four individuals suffering from macular serpiginous choroiditis. All of these eyes had a poor visual prognosis, which they attributed to foveal involvement and subsequent choroidal neovascularisation (CNV). In contrast, Sahu et al.'s 2002 report, which examined [5] nine eyes from six patients with macular serpiginous, found no evidence of CNV. Macular serpiginous choroiditis is not likely to have a higher risk of poor visual outcome than peripapillary serpiginous choroiditis as the visual prognosis in serpiginous choroiditis correlates with the closeness of the lesion to the fovea.

Serpiginous choroiditis is a rare, recurrent, progressive, and idiopathic inflammatory disease that involves the choroid and choriocapillaris and, secondarily, the retinal pigment epithelium (RPE) and retina. It affects middle-aged people, slightly more males, and it has a bilateral course. Diagnosis is most of the time based on fundus examination and fundus fluorescein angiography. Complications of untreated serpiginous choroiditis include diminution of vision secondary to macular involvement, choroidal neovascular membrane, disciform macular scarring, and so on. This article aims to present a case of tubercular serpiginous-like choroiditis that was managed in a timely manner, preventing the worsening of the condition [6-8].

## Case presentation

A healthy male in his late 30s came to the ophthalmology outpatient department with complaints of black spots in the front of both eyes and gradual, painless diminution of vision in the left eye more than the right eye, for 15-20 days. Moreover, he gave a history of left-sided sensorineural hearing loss six months back. The patient gave a history of pulmonary TB of his mother, for which she has been under treatment since the past year. His best-corrected visual acuity (BCVA) in the right eye was 20/60 with -1.50 D Cyl at 90° and 3/60 in the left eye. Intraocular pressures were normal. On a slit lamp examination, the patient had mild circumcorneal congestion in the left eye with no other findings.

On fundoscopy, grey-yellowish subretinal infiltrates at the level of the choroid, spreading centrifugally in a serpiginous (snake-like) manner in both eyes (left eye > right eye), with active scalloped edges, were seen in the central fundus (Figure 1). There was involvement of the macula in the left eye. No haemorrhages were seen in either eye. One week later, the lesions started regressing, showing a sharpening of borders with diffuse RPE mottling. There was extensive RPE atrophy. Vision in the right eye remained at 20/60, while the left eye improved to 20/400. After two months, vision improved to 20/60 in both eyes, and the patient was continued on tapering steroids while on anti-tubercular (anti-TB) drugs.

**Figure 1:** Fundus photograph showing grey-yellowish subretinal infiltrates spreading centrifugally in a serpiginous (snake-like) manner

The fundus picture seemed typical of serpiginous-like choroiditis. Fundus fluorescein angiography was performed. Renal function tests were done, and sensitivity to fluorescein was ruled out. Lesions in both eyes showed hypofluorescence with irregular and fuzzy borders in the early phase. There was leakage of the dye from choriocapillaris at the border of the inflamed lesion, and there was gradual hyperfluorescence in the mid and late phases in the right eye (Figure 2) and the left eye (Figure 3).

**Figure 2:** Fundus fluorescein angiography (right eye) showing hypofluorescent lesions in the early phase but hyperfluorescent lesions in the late phase of the angiography

**Figure 3:** Fundus fluorescein angiography (left eye) showing hypofluorescent lesions in the early phase but hyperfluorescent lesions in the late phase of the angiography

Total leucocyte count (TLC) was at 5,300/microlitre. The Mantoux test was negative. TB polymerase chain reaction (TB-PCR) (QuantiFERON gold, Cellestis Limited, Carnegie, Australia) was positive. A high-resolution CT scan of the chest was within normal limits. Serology testing for HIV, hepatitis B surface antigen (HBsAg), and hepatitis C virus (HCV) were nonreactive. The rheumatoid arthritis (RA) factor was negative.

The patient was referred to the Chest TB Department. He was started on intravenous methylprednisolone 1 g/day for three days, while on anti-TB therapy as per the directly observed treatment, short-course (DOTS) regimen:

Intensive phase (rifampicin 150 mg, isoniazid 75 mg, pyrazinamide 400 mg, ethambutol 275 mg) for two months.

Continuous phase (rifampicin 150 mg, isoniazid 75 mg, ethambutol 275 mg) for the next seven months.

After three days, he was shifted to oral steroids: tablet prednisolone 1 mg/kg body weight, amounting to 60 mg/day.

One week later, the lesions started regressing, showing a sharpening of borders with diffuse RPE mottling in the right eye (Figure 4) as well as the left eye (Figure 5). There was extensive RPE atrophy. Vision in the right eye remained at 20/60, while the left eye improved to 20/400. After one month, vision improved to 20/60 in both eyes, and the patient was continued on tapering steroids while on anti-TB drugs (Figure 6).

**Figure 4:** Right eye after a one week follow-up showing regressing lesions

**Figure 5:** Left eye after a one week follow-up showing regressing lesions

**Figure 6:** Fundus photography after one month follow-up visit showing regressing lesions

## Discussion

This was a case of choroiditis that was multifocal and bilateral in a young male. It had a snake-like morphological appearance. Serpiginous choroiditis has been considered an autoimmune disorder associated with different systemic conditions. Our patient was from a TB-endemic country, India. The TB QuantiFERON Gold was positive. Hence, the presumed diagnosis in this case is tubercular serpiginous-like choroiditis. In this patient, the lesions started in the peripapillary region and posterior pole (as against the juxtapapillary area in serpiginous choroiditis). Pigment clumping was at the centre of healed lesions (as against at the border of healed lesions in serpiginous choroiditis). Furthermore, the patient responded well to treatment with oral steroids and anti-TB drugs.

White dot syndromes are a spectrum of diseases affecting the outer retina, RPE, choroid, or a combination of these. They are multifocal and may present unilaterally or bilaterally. If present bilaterally, they are asymmetrical and also known as inflammatory multifocal chorioretinopathies. They include birdshot chorioretinopathy, acute posterior multifocal placoid pigment epitheliopathy (APMPPE), serpiginous choroiditis, relentless plaque chorioretinitis (RPC), and so on. These syndromes have no known cause and are considered autoimmune [9].

The reported prevalence of serpiginous choroiditis in patients with posterior uveitis is 5% worldwide; in India, this amounts to 19%. It was earlier known as helicoid peripapillary chorioretinal degeneration and geographical choroidopathy. It is a bilateral, recurrent, and progressive disease affecting primarily the choroid and choriocapillaris and secondarily the RPE and outer retina with disrupted flow in the choriocapillaris and inner retina, slightly more in young males compared to females. It could be an autoimmune disorder associated with systemic diseases such as sarcoidosis, Crohn’s disease, polyarteritis nodosa, systemic lupus erythematosus, non-Hodgkin’s lymphoma, and celiac disease or from an infectious aetiology such as TB, toxoplasmosis, viral infections, fungal infections, syphilis, and so on. Tubercular choroiditis could be either serpiginous-like choroiditis, or focal or multifocal choroiditis, or tuberculoma. The patient experiences a paracentral or central scotoma with vision loss. The ocular examination may show an inflammatory response in the anterior or vitreous chamber. The lesions begin in the peripapillary region or macula progressing anteriorly. Serous retinal detachment may occur in the late stages [6-8].

Because of the long-term natural history of the disease, multiple recurrences and progressive scarring lead to poor visual outcomes, and the prognosis remains poor. Hence, the goal is to prevent recurrences. Therefore, a long-term follow-up with serial fundus photographs and angiography is required to show non-progression. Fundus autofluorescence is being increasingly considered helpful [6].

The protocol for treatment focuses on systemic steroids, either oral or intravenous, depending on the severity. Intravitreal triamcinolone acetate is used where systemic steroids are contraindicated but cannot decrease recurrences. Alternative therapies include immunosuppressive drugs (i.e., cyclosporine A, azathioprine, or mycophenolate mofetil) while on anti-TB agents.

## Conclusions

Serpiginous choroiditis may affect otherwise healthy young males and can mimic other pathologies. Awareness is of utmost importance as it is a vision-threatening inflammation if not treated on time. Infective aetiologies such as TB have been commonly implicated in serpiginous-like choroiditis. Hence, proper evaluation for Koch’s aetiology with prompt treatment can prevent severe vision loss. Newer imaging techniques and newer treatment options have been rapidly emerging, but the enigma continues.
